# Correlation of Serum IGF-1R, VEGF, and ET Levels with Bone Mineral Density in Type 2 Diabetic Mellitus Patients Treated with Metformin Plus *α*-Glucosidase Inhibitors

**DOI:** 10.1155/2022/7707875

**Published:** 2022-04-21

**Authors:** Xue Chen, Xiaosheng Li, Sheng Kang, Wenbiao Duan

**Affiliations:** ^1^Department of Pathology and Pathophysiology, Zhaoqing Medical College, Zhaoqing City, Guangdong Province 526020, China; ^2^Emergency Department, Dinghu District People's Hospital, Zhaoqing City, Guangdong Province 526070, China; ^3^Department of Endocrinology, Lanling County People's Hospital, Linyi City, Shandong Province 277700, China; ^4^School Office, Zhaoqing Medical College, Zhaoqing City, Guangdong Province 526020, China

## Abstract

Diabetes mellitus is a common chronic disease. This study aimed to investigate the correlation between serum insulin-like growth factor 1 receptor (IGF-1R), vascular endothelial growth factor (VEGF), endothelin (ET) levels, and bone mineral density (BMD) in type 2 diabetic mellitus (T2DM) patients treated with metformin plus *α*-glucosidase inhibitors and evaluate the predictive value of serum factors in the prognosis of osteoporosis in these patients. It was a prospective study that enrolled 142 patients with T2DM treated in Dinghu District People's Hospital from March 2019 to May 2020. All enrollments were randomized (1 : 1) to receive either metformin (control group) or metformin plus *α*-glucosidase inhibitors (study group). After 12 weeks of treatment, metformin plus *α*-glucosidase inhibitors were associated with significantly lower levels of 2 hPG, FPG, HbA1c, and HOMA-IR versus metformin alone (*P* < 0.05). After treatment, the BMD was positively correlated with IGF-1R and negatively correlated with VEGF and ET. Alpha-glucosidase inhibitors plus metformin for primary T2DM can effectively manage blood glucose and reduce insulin resistance in patients, but the prediction of osteoporosis development remains to be further explored in large sample studies.

## 1. Introduction

Diabetes mellitus is a common chronic disease with a worldwide prevalence of about 6.4% (about 285 million patients) in 2010, and the number of cases is estimated to reach 438 million by 2030 according to the International Diabetes Federation [1–4]. Diabetes mellitus is a systemic metabolic disorder that includes abnormalities in the metabolism of sugar, lipids, protein, water, salt, electrolytes, and bone mineral. In diabetic patients, hypertonic diuresis leads to a massive loss of calcium, magnesium, and phosphorus, resulting in a decrease in bone mass and a decline in BMD due to a lack of or insufficient insulin, impaired protein anabolism, and reduced bone matrix synthesis. Metformin is currently the first choice for the treatment of type 2 diabetes mellitus (T2DM). It intensifies the body's sensitivity to insulin, boosts the utilization of glucose, lowers insulin levels, and yields a reliable hypoglycemic effect. However, some studies have indicated that the long-term use of metformin is prone to resistance and a significantly reduced hypoglycemic effect [5–7]. The *α*-glucosidase induces the conversion of starch into oligosaccharides, significantly slows down the decomposition of oligosaccharides, prevents the rapid absorption of sugars in the intestine, and decreases the postprandial blood glucose and fasting blood glucose. It also enhances insulin sensitivity and insulin resistance in the body, with a high safety profile and no drug interactions. With the aging of society and the increasing incidence of T2DM, chronic complications of diabetes mellitus have posed a great threat to diabetic patients, such as osteoporosis, severely compromising the patients' quality of life and necessitating effective prevention of OP.

Accordingly, this study investigated the efficacy of metformin plus *α*-glucosidase inhibitors on bone mineral density (BMD) in patients with T2DM and explored its mechanism of action in treating osteoporosis induced by T2DM, thereby providing references for the prevention and treatment of osteoporosis [8–11].

## 2. Materials and Methods

### 2.1. Baseline Data

It was a prospective study that enrolled a total of 142 patients with T2DM treated in Zhaoqing Medical College from March 2019 to May 2020 identified as research subjects and divided into a control group (*n* = 71) given metformin and a study group (*n* = 71) treated with metformin combined with *α*-glucosidase inhibitors. This study was approved and supported by the Ethics Committee of Zhaoqing Medical College, and the ethics approval number was 2019-2-20.

### 2.2. Inclusion and Exclusion Criteria

#### 2.2.1. Inclusion Criteria

All patients met the diagnostic criteria for T2DM: (1) fasting blood glucose (FBG) <8.88 mmol/L (160 mg/dL) for ≥1 week during hospitalization; (2) no hospital referral.

#### 2.2.2. Exclusion Criteria

The exclusion criteria are as follows: patients with allergies to the drugs used in this study; with type 1 diabetes, secondary diabetes; with concomitant endocrine system diseases; with recent use of hypoglycemic drugs; and with bone loss due to severe liver and kidney function disease and long-term bed rest.

All the included patients voluntarily participated in the study and signed the informed consent form.

### 2.3. Methods

#### 2.3.1. Medication

The control group was given oral metformin (Sino-American Shanghai Squibb Pharmaceutical Co. Ltd.; H20023370) after meals, 2 tablets/dose, three times a day. The study group was given *α*-glucosidase inhibitors (Hebei Huarong Pharmaceutical Co. Ltd.; H20103077) combined with metformin. Acarbose, 1 tablet/time, three times a day, was taken before a meal. Metformin was administered in the same way as the control group. Both groups were treated for 12 weeks [12].

#### 2.3.2. Determination of Biochemical Indexes

Before and after treatment, five mL of morning fasting venous blood was collected from all patients and centrifuged to obtain the serum. The serum was divided into two samples. One sample was used to determine FPG, and hemoglobin A1c (HbA1c) levels in both groups using a Roche automatic biochemical analyzer. The other sample was frozen at −70°C for the determination of serum insulin-like growth factor 1 receptor (IGF-1R), vascular endothelial growth factor (VEGF), endothelin (ET), and bone alkaline phosphatase (B-ALP) levels using the double antibody sandwich enzyme-linked immunosorbent assay (ELISA). Before and after treatment, five mL of venous blood was also collected at 2 hours after a meal and centrifuged to obtain the serum, and the level of 2-hour postprandial blood glucose (2 hPG) was determined using the Roche automatic biochemical analyzer [13, 14]. BMD measurement: the BMD of the lumbar spine 1–4 (L1–4), femoral neck (FN), and total hip (TH) of the patients were measured using a LunarDPX-NT dual-energy X-ray absorptiometry (DXA), manufactured by GE, USA [15, 16].

### 2.4. Statistical Analyses

Data analysis was performed using SPSS 22.0. The measurement data were expressed as ($\bar{x}$ ± *s*) using the *t*-test, the count data were expressed as percentages (%) and processed by the chi-square test, and the correlation analysis was performed using Pearson correlation analysis. A difference was considered statistically significant at *P* < 0.05.

## 3. Results

### 3.1. Baseline Data

The control group had 39 males and 32 females, aged 43–71 years, with a mean age of (56.62 ± 8.14) years, a mean BMI (22.49 ± 3.62) kg/m^2^, mean duration of disease of (10.67 ± 8.01) years; 43 cases had a history of drinking, and 44 had a history of smoking. The study group had 34 males and 34 females, aged 44–73 years, with a mean age of (57.17 ± 8.73) years, a mean BMI (22.99 ± 3.83) kg/m^2^, and mean duration of disease of (10.25 ± 7.49) years; 42 cases had a history of drinking, and 46 had a history of smoking. The two groups showed no significant difference in baseline data (*P* > 0.05) (see Table 1).

### 3.2. Blood Glucose-Related Indexes

Before treatment, the serum levels of FPG, 2 hPG, HbA1c, and HOMA-IR were comparable between the two groups. After treatment, the above indicators were lower in the study group (all *P* < 0.05). Metformin plus *α*-glucosidase inhibitors were associated with significantly lower levels of HbA1c, FPG, 2 hPG, and HOMA-IR in patients with T2DM versus the single-use of metformin (*P* < 0.05). (Table 2).

### 3.3. Bone Metabolic Indexes

After treatment, the bone gal protein (BGP) levels decreased in both groups and the blood calcium and blood phosphorus levels showed no significant changes. After treatment, alkaline phosphatase (ALP) and parathyroid hormone (PTH) levels were increased and urinary cyclophosphamide (CTX) levels were decreased in both groups, as shown in Table 3.

### 3.4. Serum Factors and BMD

The post-treatment IGF-1R level was significantly increased and was positively correlated with BMD (*r* = 0.142), while the post-treatment VEGF level was significantly decreased and was negatively correlated with BMD (*r* = −0.05) (Figures 1–3). After treatment, the ET level was significantly reduced and was negatively correlated with BMD (*r* = −0.051), as shown in Table 4.

## 4. Discussion

The results of the present study showed that metformin plus *α*-glucosidase inhibitors were associated with significantly lower levels of HbA1c, FPG, 2 hPG, and HOMA-IR in patients with T2DM versus the single-use of metformin (*P* < 0.001), suggesting a stronger hypoglycemic effect of the joint use of drugs than single medication [17, 18]. The role of cytokines in the pathogenesis of osteoporosis can be observed by investigating the correlation between relevant factors and BMD after medication of metformin plus *α*-glucosidase inhibitors. The results demonstrated that blood glucose-related indexes were significantly reduced after treatment, and serum IGF-1R was positively correlated with lumbar spine BMD (*r* = 0.142, *P*=0.119), presumably because the HbA1c content reflects the blood glucose content within a certain period, and the reduction of blood glucose after treatment promotes the synthesis and release of IGF-1R, which accelerates the replication of osteoblasts and the formation of bone matrix and increases the deposition of calcium and collagen synthesis in bones, thus increasing the bone density. Moreover, VEGF was negatively correlated with lumbar spine BMD after treatment (*r* = −0.05, *P*=0.341). VEGF may be involved in bone formation and angiogenesis and be closely related to bone metabolism and bone conversion, so it is considered an important factor in the pathophysiological process of diabetic osteoporosis. ET is a vasoactive factor with a strong vasoconstrictive effect, which is intimately associated with cardiovascular and cerebrovascular diseases and involved in the development of osteoporosis. In the present study, after treatment, the serum ET level was negatively correlated with lumbar spine BMD (*r* = −0.051, *P*=0.338) and IGF-1R (*P* < 0.05), which is attributable to the inhibition of ET expression after the increase of IGF-1R. The study by Qin et al. indicated a negative correlation between ET-1 and IGF-1R in coronary artery disease and a mutual influence of the two in the progression of the disease [19–22].

## 5. Conclusion

Alpha-glucosidase inhibitors plus metformin for primary T2DM can effectively manage blood glucose and reduce insulin resistance in patients, but the prediction of osteoporosis development remains to be further explored in large sample studies.

## Figures and Tables

**Figure 1:** Correlation between IGF-1R and lumbar BMD.

**Figure 2:** Correlation between VEGF and lumbar BMD.

**Figure 3:** Correlation between ET and lumbar BMD.

**Table 1:** Comparison of baseline data.

Groups	Study group	Control group	$\bar{x}$ /*t*	*P* value
*n*	71	71		
Gender (male/female)	39/32	37/34	0.113	0.736
Age				
Range	43∼71	44∼73		
Mean age	56.62 ± 8.14	57.17 ± 8.73	0.388	0.699
Mean BMI	22.49 ± 3.62	22.99 ± 3.83	0.799	0.426
Mean course of disease	10.67 ± 8.01	10.25 ± 7.49	0.323	0.747
Drinking	43	42	0.029	0.864
Smoking	44	46	0.121	0.728

**Table 2:** Comparison of FPG, 2 hPG, HbA1c, and HOMA-IR levels.

Groups	*n*	FPG (mmol/L)		HbA1c (%)		2 hPG (mmol/L)		HOMA-IR	
		Before treatment	After treatment	Before treatment	After treatment	Before treatment	After treatment	Before treatment	After treatment
Study group	71	9.48 ± 2.34	6.12 ± 1.03^a^	9.23 ± 1.29	6.55 ± 2.03^a^	13.54 ± 2.83	7.13 ± 3.02^a^	5.27 ± 1.09	2.65 ± 0.82^a^
Control group	71	10.13 ± 1.71	6.89 ± 0.95^a^	8.87 ± 1.57	7.54 ± 1.74^a^	13.63 ± 2.07	10.26 ± 2.33^a^	5.14 ± 1.03	3.46 ± 1.01^a^
*t*		1.89	4.63	1.493	3.12	0.216	6.914	0.73	5.246
*P* value		0.061	<0.001	0.138	0.002	0.829	<0.001	0.467	<0.001

^a^Post-treatment compared with pretreatment, *P* < 0.05.

**Table 3:** Comparison of bone metabolic indexes.

Groups	*n*	BGP		Blood calcium		Blood phosphorus		ALP		PTH		Urinary CTX	
		Before treatment	After treatment	Before treatment	After treatment	Before treatment	After treatment	Before treatment	After treatment	Before treatment	After treatment	Before treatment	After treatment
Study group	71	13.44 ± 2.64	22.47 ± 5.37	2.48 ± 0.12	2.49 ± 0.13	1.26 ± 0.26	1.23 ± 0.26	75.31 ± 21.34	86.94 ± 27.35	28.24 ± 8.34	36.42 ± 17.36	917.10 ± 451.65	460.27 ± 180.63
Control group	71	13.67 ± 2.57	15.32 ± 3.76	2.47 ± 0.11	2.45 ± 0.15	1.25 ± 0.12	1.22 ± 0.12	74.62 ± 27.69	80.62 ± 27.69	28.59 ± 8.19	49.37 ± 15.36	916.87 ± 449.87	554.38 ± 361.53
*t*		0.139	9.19	0.518	1.698	0.294	1.471	0.166	1.368	0.252	4.708	0.003	7.441
*P* value		0.89	<0.001	0.605	0.092	0.769	0.144	0.868	0.173	0.801	<0.001	0.998	<0.001

**Table 4:** Comparison of serum factors and BMD.

Groups	*n*	IGF-1R (ng/mL)		VEGF		ET (pg/mL)		BMD (g/cm^2^)	
		Before treatment	After treatment	Before treatment	After treatment	Before treatment	After treatment	Before treatment	After treatment
Study group	71	145.31 ± 17.23	194.27 ± 22.61^a^	217.72 ± 48.37	195.77 ± 50.24^a^	93.65 ± 13.96	61.80 ± 10.39^a^	0.88 ± 0.03	1.26 ± 0.09^a^
Control group	71	146.74 ± 17.86	170.22 ± 18.52^a^	218.41 ± 50.22	178.34 ± 45.27^a^	94.04 ± 12.78	73.75 ± 11.73^a^	0.87 ± 0.05	1.14 ± 0.07^a^
*t*		0.486	6.934	0.083	2.172	0.174	6.426	1.445	8.868
*P* value		0.628	<0.001	0934	0.032	0.862	<0.001	0.151	<0.001

^a^Post-treatment compared with pretreatment, *P* < 0.05.

## Data Availability

The datasets used during the present study are available from the corresponding author upon reasonable request.
